The article "Individualistic sensitivities and exposure to climate change explain variation in species’ distribution and abundance changes" was retracted in 2016. Reasons: errors in the materials; errors in the methods; unreliable results or conclusions.

# Individualistic sensitivities and exposure to climate change explain variation in species’ distribution and abundance changes

**DOI:** 10.1126/sciadv.1400220

**Published:** 2015-10-30

**Authors:** Georgina Palmer, Jane K. Hill, Tom M. Brereton, David R. Brooks, Jason W. Chapman, Richard Fox, Tom H. Oliver, Chris D. Thomas

**Affiliations:** 1 Department of Biology, University of York, Wentworth Way, York YO10 5DD, UK.; 2 Butterfly Conservation, Manor Yard, East Lulworth, Wareham, Dorset BH20 5QP, UK.; 3 AgroEcology Department, Rothamsted Research, Harpenden, Hertfordshire AL5 2JQ, UK.; 4 Environment and Sustainability Institute, University of Exeter, Penryn, Cornwall TR10 9EZ, UK.; 5 NERC (Natural Environment Research Council) Centre for Ecology and Hydrology, Benson Lane, Crowmarsh Gifford, Oxfordshire OX10 8BB, UK.

**Keywords:** environmental change, extinction, sensitivity, Lepidoptera, population dynamics, anthropocene, colonisation, range shifts, climatic variability, biogeographic responses

## Abstract

The responses of animals and plants to recent climate change vary greatly from species to species, but attempts to understand this variation have met with limited success. This has led to concerns that predictions of responses are inherently uncertain because of the complexity of interacting drivers and biotic interactions. However, we show for an exemplar group of 155 Lepidoptera species that about 60% of the variation among species in their abundance trends over the past four decades can be explained by species-specific exposure and sensitivity to climate change. Distribution changes were less well predicted, but nonetheless, up to 53% of the variation was explained. We found that species vary in their overall sensitivity to climate and respond to different components of the climate despite ostensibly experiencing the same climate changes. Hence, species have undergone different levels of population “forcing” (exposure), driving variation among species in their national-scale abundance and distribution trends. We conclude that variation in species’ responses to recent climate change may be more predictable than previously recognized.

## Teaser

Analysis of butterfly and moth species shows that responses to climate change may be more predictable than previously recognized.

## INTRODUCTION

Species’ responses to recent environmental changes have been highly heterogeneous, showing a diversity of trends in abundances, overall geographic range sizes, latitudinal and elevational positions, dynamics of range boundaries, and directions of range shifts (*1*–*7*). The magnitude of variation among individual species is greater than the average magnitude of the changes (*2*), consistent with the individualistic responses of species to climatic changes during the Pleistocene glacial and interglacial cycles (*8*–*10*). The limited success of attempts to explain this high interspecific variation implies a fundamental lack of understanding about how drivers of change operate and how species respond to these climate changes (*4*). Here, we attempt to explain the variation in species’ responses to climate.

When the climate warms, species are widely assumed to experience an improvement in climatic conditions at the cool edges of their ranges, resulting in increased abundances and larger regional distribution sizes (*6*, *8*, *11*–*13*). Yet, empirical data suggest that the range expansions of some species apparently exceed the rates of climate warming, whereas other species have decreased their ranges when they have been expected to increase (*2*, *3*, *6*, *14*). If complex and interacting biological and environmental processes are the main determinants of change, it may therefore be difficult to predict future responses to climate change. Alternatively, the diverse ways in which species respond may arise from individualistic responses to the climate itself, making predictions more straightforward.

Many studies have described the relationships between climate and species’ population dynamics [see the work of Parmesan (*15*) for a review]. In general, such studies highlight the individualistic responses of species to climate and conclude that some species are more sensitive to climate than others. For example, Roy *et al*. (*16*) described the relationships between climate and the abundance of 31 British butterflies (17 of which are also included in our analyses). They found considerable variation in the climate variables that species were influenced by, as well as some species being much more sensitive to climate than others. However, sensitivity alone does not capture species’ response to climate change, because a species may be sensitive to several components of climate but may not be exposed to changes in those climate components. For example, a species could be sensitive to summer precipitation, but the predominant locally occurring climatic change the species is exposed to is an increase in spring and autumn temperatures. Both climate sensitivity and exposure have been described and quantified by a number of authors (*17*–*19*), and these studies have shown that species vary in both their sensitivity and exposure to climate change, that sensitivity and exposure are not necessarily correlated, and that both sensitivity and exposure are important factors in describing species’ vulnerability to climate change. However, the terms “sensitivity” and “exposure” have not been used consistently in the literature. Some authors regard sensitivity to be an attribute of a species, independent of local climate conditions, and exposure to be solely a measure of climate change. We argue instead that sensitivity and exposure emerge from the interaction between an organism and the climate and should not be separated into species-only and environment-only components. Thus, the sensitivity of a species needs to be considered in the context of the climatic variability that the species experiences and the exposure experienced by a species in the context of longer-term changes in those components of climate to which the species is responsive.

Here, we test the hypothesis that variation in the observed responses of species to recent climate change is predominantly because species vary in how they are affected by climate (that is, differences in their sensitivity and exposure to climate). Specifically, we investigate variation in three commonly studied responses of species—changes in abundance, changes in distribution size, and changes in the northern range margin location (*20*). We examine whether variation among species in these responses can be explained by differences in their sensitivity and exposure to climate change (Fig. 1). We measure the sensitivity of species as the extent to which year-to-year changes in abundance over four decades are explained by seasonal temperature and rainfall variables. Our measure of sensitivity varies from 0 when none of the year-to-year abundance changes can be explained by temperature and rainfall variables, to a value of 1 when 100% of the variation is explained. Exposure is more complex to compute because different species are sensitive to different components of the climate (that is, responding positively or negatively to precipitation and/or temperature at different times of year), which will have changed to different extents over the four decades of our study. We measure the exposure of each species on the basis of the climate variables to which it is individually sensitive. Our exposure values are negative if the climate that a species is sensitive to drives population decline and positive when the climate drives population growth. Exposure is measured on a log scale, so a value of +0.69 represents a climate-driven mean doubling of populations annually, whereas a value of −0.69 represents a climate-driven mean annual decrease of 50%. Our measures of sensitivity and exposure are both computed from the analysis of interactions of species with climate, and thus are not independent of each other, but measures of sensitivity and exposure are not necessarily correlated with one another (below). There is also no necessary analytical reason why sensitivity and exposure should be correlated with long-term abundance and distribution changes if there is no temporal trend in the seasonal climate conditions to which a species is sensitive, or if nonclimatic factors ultimately limit species’ abundances and distributions.

**Fig. 1:** Flowchart of methodological approach. Species-specific climate models were built by relating year-to-year changes in relative abundance to seasonal climate variables. Species-specific sensitivity and exposure metrics were derived from the outputs of the species-specific climate models and were used as predictor variables in models explaining interspecific variation in changes in species’ abundance, distribution size, and northern range margins.

We test our hypothesis by studying 155 species of Lepidoptera (24 butterflies and 131 macromoths; table S1) in Great Britain (GB), an exemplar group with the most complete species-specific population and distributional data for any poikilothermic animal group in the world (~26 million distribution records and ~34 million individuals counted in light traps or along transects across GB). These data are unrivalled in terms of our capacity to evaluate the sensitivity of species to climatic variation and to quantify the exposure of species to more than four decades of climate change. All of the study species are southerly distributed, with a northern (in principle leading-edge) range limit within northern Britain. These species have hitherto been assumed to respond positively to regional warming (*6*, *13*, *14*, *21*), given their historical restriction to warmer parts of Britain. Hence, it might be expected that all of these study species would increase in abundance, expand their ranges, and shift their range boundaries northward in GB in response to climate warming, assuming that suitable habitats are available within their dispersal range (*22*, *23*). However, in reality, these species have shown considerable variation in their abundance (*1*, *13*, *14*) and distribution (*2*, *6*, *14*) trends (Fig. 2) over the past four decades of climate change. Here, we assess the degree to which species’ sensitivity and exposure can explain this variation in species’ responses to recent climate change (Fig. 1).

**Fig. 2:** Responses of species to climate change. (**A** to **C**) Frequency distributions of changes in (A) abundance, (B) distribution size, and (C) northern range margin of butterflies (dashed bars, *n* = 24 species) and moths (open bars, *n* = 131 species). Changes in distribution size and northern range margin were calculated using well-recorded hectads. In each plot, values for each taxonomic group were standardized so that mean = 0 and variance = 1.

## RESULTS

To examine interspecific variation in species’ sensitivity to climate, we first quantified how variation in seasonal temperature and rainfall affected year-to-year changes in species’ relative abundances over the past four decades (1968–2012 for moths, 1976–2012 for butterflies). Year-to-year changes in the abundances of each of our 155 species were analyzed in relation to seasonal measures of temperature and rainfall (four seasons and annual lagged effects; see table S2 for a full description of variables). In total, 94 species (61%) responded to both temperature and rainfall variables, 36 (23%) responded only to temperature variables, and 25 (16%) only to rainfall variables (table S1). There were no consistent patterns in which seasonal climate variables influenced the population dynamics of our study species or in the importance and direction of their effects (table S1, Fig. 3D, and fig. S1).

**Fig. 3:** Variation in species’ sensitivity and exposure to climate change, and the aspects of the climate they are most sensitive to. (**A** to **D**) Frequency distributions of butterfly (dashed bars, *n* = 24 species) and moth (open bars, *n* = 131 species) sensitivities (A) and exposures (B) to climate, the relationship between exposure and sensitivity (C), and climate variables in species’ climate models (D). Sensitivity is the proportion of year-to-year change in a species’ population trend that can be attributed to variation in the climate. Exposure represents the mean annual change in these population trends (+, predicted increase; −, predicted decrease) expected for each species on the basis of 1970–2010 climatic conditions and the climate variables to which each species is sensitive. (C) There was no significant relationship between species’ climate sensitivity and exposure (Spearman’s *r* = 0.02, *P* = 0.82). (D) Variables represent either the sum of rainfall (white boxes) or mean temperatures (gray boxes) for a given season [spring (March–May), summer (June–August), autumn (September–November), or winter (December–February)] in the current year (“year *t*”), the previous year (“year *t*−1”), or 2 (“year *t*−2”) or 3 years previously (“year *t*−3”). Variables were standardized before analysis. The numbers of species in each column are provided in bold italic font above the *x* axis—each species’ best climate model contained up to three climate variables, and therefore, each species is represented in up to three columns. Medians are represented by the horizontal black lines; the top and bottom of each box are the 75th and 25th percentiles, respectively; outliers are represented by black dots; and whiskers represent data within 1.5 × interquartile range (IQR) of the upper and lower quartiles.

### Species’ sensitivity to climate change

We quantified the sensitivity of each of our study species according to the amount of variation in year-to-year abundance changes explained by the climate variables to which they were most responsive (climate models included a maximum of three variables per species; Eq. 1 and Materials and Methods). Year-to-year abundance changes of some species were strongly explained by seasonal climate variables (that is, *R*^2^ values of climate models were high), whereas others were only weakly explained (Fig. 3A). Thus, our measure of species’ sensitivity varied from 0.09 for the northern winter moth *Operophtera fagata*, to 0.82 for the shuttle-shaped dart moth *Agrotis puta* (mean sensitivity across all 155 species, 0.45 ± 0.01 SE; Fig. 3A).

### Species’ exposure to climate change

The diversity of species’ sensitivity to temperature and rainfall variation demonstrates that individual species also varied in their exposure to climate change (Fig. 3B). We measured exposure using the individual species’ climate models (Eq. 1 and table S1) in combination with climate data from 1970 to 2010 to quantify the direction and magnitude of expected annual population change as a result of variation in those aspects of climate to which each species is most responsive. Among the 155 study species, exposure varied from −0.15 (equivalent to a mean yearly decline of 14%) for the white admiral butterfly *Limenitis camilla*, to +0.18 (equivalent to a mean yearly increase of 20%) for the orange-tip butterfly *Anthocharis cardamines*. A total of 77 (50%) species experienced positive exposure (≥0), that is, climate to which those species were responsive to improved, whereas 78 (50%) species experienced negative exposure (exposure < 0), that is, climate to which those species were responsive to deteriorated. Mean exposure across all 155 species was −0.01 ± 0.004 SE (equivalent to a mean decline of 1% per year; Fig. 3B).

Our measures of species-specific exposure and sensitivity are derived from the same data sets but are not correlated (Spearman’s *r* = 0.02, *P* = 0.82; Fig. 3C). Thus, a climate-sensitive species that has a high percentage of year-to-year abundance changes—explained by seasonal temperature and rainfall variables—does not necessarily experience long-term beneficial or detrimental (in terms of population impact) trends in the climate to which it is sensitive. For example, the ringlet butterfly *Aphantopus hyperantus*, the dusky thorn moth *Ennomos fuscantaria*, and the small dusty wave moth *Idaea seriata* are all highly sensitive to yearly variation in the climate, with sensitivities of 0.69, 0.74, and 0.79, respectively. However, the ringlet has experienced relatively high positive exposure (0.12; maximum value across all species, 0.18), whereas the dusky thorn moth has experienced negative exposure (−0.07; minimum value across all species, −0.15) and the small dusty wave has experienced little exposure (−0.009). Thus, these three species have experienced improving climate (ringlet), deteriorating climate (dusky thorn), and little change in the climate (small dusty wave) despite all of them occupying the same geographic region, ostensibly experiencing the same climate conditions, and being similarly sensitive to climate.

### Explaining variation in species’ responses to climate

Once we had quantified the sensitivity and exposure of species, we then examined whether these two measures explained the variation in species’ responses to climate in terms of their abundance and distribution trends. We quantified the changes in species’ abundances (as the slope of long-term population trend), overall distribution sizes (change in areal extent; GB Ordnance Survey grid; 10 km hectads decade^−1^), and northern range margins (km shift north decade^−1^). These variables were obtained from the distribution and count (transect and light-trap data) records of butterflies and macromoths from within our study area (fig. S2), collected between ~1970 and 2010 (see Materials and Methods). Species demonstrated considerable variation in changes in their distribution sizes [median (IQR), +77.6 hectads decade^−1^ (−34.8, 107.8)], northern range margins [12 km shift north decade^−1^ (−39.2, 21.0)], and abundances [slope of long-term abundance trend, −0.02 (−0.07, 0.02)] (Fig. 2).

Species’ exposure and, to a lesser extent, sensitivity were strong predictors of the long-term abundance trends of butterflies and moths (Fig. 4, A and B). A total of 64 and 59% of variation in the long-term abundance trends of butterflies and moths, respectively, could be explained by their exposure to climate change (for moths) or by a positive interaction between their exposure and sensitivity (for butterflies) (Table 1). Exposure and sensitivity also predicted, but less strongly, changes in the distribution sizes of study species. Thus, 53% of the variation in butterfly range size changes was explained by their sensitivity and exposure to climate (Fig. 4C), whereas 22% of the variation in moth range size changes was explained by their exposure to climate (Fig. 4D). By contrast, only 14% of the variation in range margins shifts could be explained by butterfly species’ exposure to climate change, and 3% could be explained for moths (Table 1 and Fig. 4, E and F).

**Fig. 4:** Species’ distribution and abundance changes related to their sensitivity and exposure. (**A** to **F**) Relationships between changes in the abundance (A and B), distribution size (C and D), and northern range margin (E and F) of butterflies (*n* = 24) and moths (*n* = 131) in relation to either their exposure to climate change (B, D, E, and F) or the interaction between exposure and sensitivity to climate change (A and C). The proportions of variation explained by each model (A to F) were 0.64, 0.59, 0.53, 0.22, 0.14, and 0.03, respectively. For (B), (D), (E), and (F), modeled relationships (solid lines) ± SE (dashed lines) are depicted; for (A) and (C), modeled relationships between response variables and climate exposure are shown, with sensitivity values kept constant [at the observed minimum (−2.29; short-dashed line), mean (0.00; solid line), and maximum (1.98; long-dashed line) sensitivity values]. All variables were standardized so that mean = 0 and variance = 1.

**Table 1:** Candidate models (within 2 AIC units of the best model) for multivariate regressions relating response variables to the sensitivity (“Sens”) and exposure (“Exp”) of butterflies (*n* = 24) and moths (*n* = 131) to climate. SEs are provided within brackets; bold values indicate individually significant effects. Response variables were standardized values of changes in abundance, distribution size, and northern range margin; the latter two variables were calculated using well-recorded 10 × 10–km grid squares (hectads) and standardized before analysis to enable comparisons between the size and direction of coefficients.

**Response**	**Taxa**	**Intercept**	**Exposure**	**Sensitivity**	**Exp:Sens**	**ΔAIC**	***R*^2^**
Δ Abundance	Butterfly	−0.05	**0.68 (0.12)**	0.16 (0.14)	**0.35 (0.14)**	0.00	0.64
	Moth	0.29	**0.80 (0.07)**			0.00	0.59
Δ Distribution size	Butterfly	0.56	**0.63 (0.28)**	0.20 (0.24)	0.26 (0.33)	0.00	0.53
	Butterfly	1.31	**0.66 (0.12)**			0.13	0.45
	Moth	0.00	**0.45 (0.07)**			0.00	0.22
Δ Northern range margin	Butterfly	−0.37	0.25 (0.13)			0.00	0.14
	Butterfly	−0.40				1.58	0.00
	Moth	−0.10	**0.22 (0.06)**			0.00	0.03
	Moth	−0.15	0.08 (0.06)	−0.03 (0.06)	**−0.15 (0.06)**	1.89	0.05

## DISCUSSION

Despite species, on average, shifting their distributions in the direction expected with the observed climate change (*2*), there remains considerable unexplained variation in their abundance and distribution trends (Fig. 2), which is most frequently interpreted as being associated with nonclimatic factors. However, we found that a high proportion of this between-species variation could be explained by species-specific exposure and sensitivity to climate. In particular, abundance changes were particularly strong for climate-sensitive butterfly species that were positively exposed to the highest levels of climatic change (Fig. 4A). Although moths were apparently more affected by their exposure to climate than by their sensitivity, our measure of exposure represents the interaction between intrinsic (the variables to which a species is sensitive) and extrinsic (changes in those climate variables) factors. Hence, we conclude that more than half of the variation in national-scale abundance changes of these southerly distributed species could be explained by climatic-associated population “forcing” since the 1970s, as experienced individualistically by each species. Associations between sensitivity, exposure, and long-term abundance trends are not inevitable, even though we used abundance data to compute year-to-year changes in species’ relative abundance, which are incorporated into species-specific climate models, as well as to compute species’ responses to climate, on the basis of species’ long-term abundance trends over four decades. We do not necessarily expect associations because each species’ climate model is based on one species, and this does not inevitably lead to high predictive power when estimating the differences between species. More importantly, had the total abundances (equivalent to local carrying capacities) of these species been set by nonclimatic factors, a series of climatically favorable or unfavorable years (as deduced by the models) would not result in the long-term changes in abundance that were observed over the entire period. For example, Pateman *et al*. (*24*) found that long-term positive abundance changes were not achieved by the brown argus butterfly *Aricia agestis*, despite a favorable climate (that is, positive exposure), because abundances were limited by other nonclimatic factors.

We had assumed that our southerly distributed poikilothermic study species might have benefited from climate warming over the past four decades, but unexpectedly, half of our 155 study species experienced negative exposure (that is, the climate deteriorated for them) over a period when UK mean temperatures during the boreal summer increased by 1.15°C (UK Met Office data). Thus, the observed climate changes were not favorable for all of our species. This unexpected finding is partly attributable to the fact that although 53 species responded positively to warm conditions in the current summer, most of the 48 species that responded to temperature in the previous summer did so negatively (Fig. 3D and fig. S1). These lagged effects from previous years may be caused by climate-driven changes in biotic interactions with host plants, competitors, and natural enemies (*24*, *25*). However, the exposure of species was not linked to species’ sensitivities to one or a few specific climate variables because there was no overall difference in the most versus least exposed species with respect to the strength of their responses to either temperature or precipitation (Fig. 3D, fig. S1, and table S1). Thus, some species were more sensitive to precipitation, others to temperature, but with no evidence that this was linked to overall sensitivity or exposure (table S1). Even if species responded to the same climatic variables, they often did so in opposite directions, in different seasons, and to climate in different years (that is, lagged effects associated with conditions in the preceding year versus current year direct effects; Fig. 3D, fig. S1, and table S1). As with similar studies of our study taxa [for example, the study of Roy *et al*. (*16*)], species were consistently inconsistent with respect to their responses to climate change.

On the basis of the distribution and abundance changes that we investigated, we found that species’ sensitivity and exposure best predicted national-scale abundance changes, rather than changes in geographic range sizes (*12*, *26*) or northern range margin shifts. This is likely to be due to the imperfect correlation between abundance changes and range size and margin changes (*1*, *14*), variation in dispersal and habitat availability (required for colonization and persistence), and lag times and nonequilibrium distribution patterns. The nature of the data used to estimate abundance and distribution changes was also different. Nevertheless, 53% of the variation in butterfly distribution changes and 22% of the variation in moth distribution changes could be explained by their species-specific exposure and sensitivity to climate, with positively exposed species showing the highest increase in distribution size over our period of study.

Compared with the other responses we examined, variation in the northward (poleward) range margin shifts of species was least well predicted by exposure and sensitivity, reflecting the large sample errors associated with estimating range margin locations (*27*). In addition, the wide range of climatic sensitivities and exposures of the study species may not necessarily result in north-south distribution changes (*28*). For example, species responding to rainfall might be expected to shift east-west in Britain. The explanatory power of our different models (abundance > distribution size > northern range margin variation) suggests that responses to climate change are better understood by large-scale population monitoring programs than by recording range size changes or boundary shifts with the methods used in this and other studies (*12*, *26*, *27*), at least in the high-latitude regions of species’ distributions. Distribution data can provide valuable insights into broad patterns of responses (particularly when averaged across species), but monitoring data seem better suited to detect the specific role of climate in these trends.

In conclusion, about 60% of the between-species differences in abundance trends were attributable to their species-specific exposure and sensitivity to climate, suggesting that variation in species’ responses to recent climate change may be more predictable than previously recognized. Our study focuses on explaining variation in the distributions and abundances of species in the northern (coolest) parts of their ranges, and further research is required to evaluate whether populations of the same species in different regions will show the same responses to climate (*29*). The widely held assumption that late 20th and early 21st century warming would have improved conditions for species in the coolest parts of their distributions was not supported for many species. Species responded differently to the same climatic changes, and many southerly species experienced deterioration, rather than improvement, in climate conditions. Individualistic responses to recent climate are already under way and are likely to cause non-analog ecological communities to emerge (*30*, *31*).

## MATERIALS AND METHODS

### Experimental design

We examined causes of variation in the responses of 155 British butterfly and macromoth species to recent climate change. First, we built species-specific climate models to determine their sensitivity and exposure to climate. We then quantified responses of species to climate change using three commonly used metrics: change in abundance, change in distribution size, and change in northern range margin location. Finally, we examined how much of the variation in species’ responses to recent climate change could be explained by differences in species’ sensitivity and exposure. In the methods, we describe (i) the sources of data that we analyze; (ii) our species-selection criteria; (iii) the generation of species-specific climate models; (iv) our measures of sensitivity and exposure; (v) how we quantify species’ responses to climate in relation to changes in abundance, range size, and range margin location; and (vi) how we relate variation among species in their responses to climate to their species-specific sensitivity and exposure (Fig. 1).

**Sources of data.** Two types of data for Lepidoptera were analyzed: data on abundance from long-running transect and light-trap surveys and data on distributions. We describe these data below.

*Abundance data*: Count data for butterflies from 2105 sites spanning the years 1976–2012 and for moths from 425 sites spanning the years 1968–2012 were obtained from the UK Butterfly Monitoring Scheme (UKBMS transects) and the Rothamsted Insect Survey (RIS light-trap surveys), respectively. We defined our study area as mainland GB and islands within 10 km of the mainland; all data were within this geographic boundary. Not all sites have data for every year and not all species occur on every site [number of sites per species, 314 ± 23 (mean ± SE)]. The UKBMS and RIS are national networks of standardized count surveys for Lepidoptera and have been running since 1976 and 1968, respectively. Although different methods are used in these two schemes—walking transects for butterflies and light traps for moths—the abundance data collected are comparable and have previously been used to calculate collated indices of abundance for species within both taxonomic groups (*13*, *32*, *33*).

These abundance data were used in two different ways. First, year-to-year changes in abundance were used as the response variable in species-specific climate models (Fig. 5, C and D), which were then used to quantify species’ sensitivity and exposure to climate change. Second, abundance data were used to compute long-term abundance trends (Fig. 5, C and D). However, as mentioned in Discussion, there is no need for year-to-year changes in abundance to relate to long-term abundance trends.

**Fig. 5:** Population changes of two exemplar butterfly species. (**A** to **H**) Distributions, abundance trends, exposure, and sensitivities of two exemplar butterfly species: the comma *Polygonia c-album* (A, C, E, and G) and the grizzled skipper *Pyrgus malvae* (B, D, F, and H). (A and B) Distribution changes between 1970–1985 and 1995–2010. Black squares are well-recorded hectads occupied in both time periods, gray squares are those colonized by the second period, and red squares show locations of apparent extinctions. Northern range margins in the first and second time periods are represented by the dashed and horizontal lines, respectively. (C and D) Observed log collated indices of abundance (solid lines) and the modeled linear change in the index (dashed lines); the slope of this relationship is defined as species’ long-term change in abundance. (E and F) Observed (black lines) and predicted (red lines) change in log collated index; sensitivity represents the proportion of year-to-year change in a species index of abundance that can be attributed to variation in the climate (that is, *R*^2^), and exposure is calculated as the predicted mean annual change in index between 1970 and 2010. Predicted changes in index were calculated using climate models with coefficients depicted in (G) and (H).

*Distribution data*: Butterfly and macromoth distribution records from within our study area for the periods 1970–1985 and 1995–2010 were obtained from the National Moth Recording Scheme (NMRS) (*34*) and the Butterflies for the New Millennium (BNM) (*35*) recording schemes run by Butterfly Conservation. These data comprise spatially and temporally explicit species observations collated opportunistically by recorders from field surveys (for all life stages) and light-trapping. For this analysis, each record was attributed to the hectad (10 × 10–km grid square) of the Ordnance Survey National Grid in which it occurred. These distribution data were used to quantify responses to climate change (changes in distribution size and changes in northern range margin).

*Climate data*: Monthly data representing mean temperature (°C) and sum of precipitation (mm) at a 5 × 5–km grid resolution across our GB study area for the years 1966 to 2011 were obtained from the UK Met Office (UKCP09; www.metoffice.gov.uk/climatechange/science/monitoring/ukcp09; data for 2012 were not yet available). These data were grouped into 3-month blocks corresponding to boreal autumn (September, October, and November), winter (December, January, and February), spring (March, April, and May), and summer (June, July, and August). Seasonal mean temperatures and sum of rainfall were calculated for each 5-km grid square. We then calculated annual mean values per season for the GB study area. Climate data were standardized (so that $\bar{x}$ = 0 and variance = 1) before analysis so that the relative importance of the variables could be assessed in statistical models. Absolute correlation between all combinations of climate variables did not exceed 0.58 [absolute Pearson’s correlation coefficient = 0.16 ± 0.13 (mean ± SD); table S2].

**Species selection criteria.** We analyzed data for 24 butterfly and 131 macromoth species that reach their northern range margins in GB (that is, southerly distributed species; table S1). Species were excluded if their northern range boundary in the first time period (see next section) was within 100 km of the northern limits of the study area [the maximum range shift recorded previously (*6*) to avoid geographical truncation of observed range shifts]. We also excluded species for which the mean altitude of occupied hectads in the first time period was more than 200 m (that is, excluding montane species that may shift altitudinally rather than latitudinally). For inclusion, species also needed to be recorded in 20 or more hectads in the first period and to be present in both time periods so that changes in distribution could be calculated [following Thomas and Lennon (*36*)]. Species were also excluded if they were migrants or underwent taxonomic revision since 1968, or if abundance data were not available to make reliable long-term population trend estimates (requiring at least five transect/light-trap sites in every year).

**Species-specific climate models.** To calculate species-specific sensitivity and exposure metrics, we first modeled how variation in seasonal temperature and rainfall affected year-to-year changes in species’ relative abundances over the past four decades (1968–2012 for moths, 1976–2012 for butterflies). Year-to-year changes in the abundances of each of our 155 species were analyzed in relation to 24 seasonal measures of temperature and rainfall (four seasons, and annual lagged effects, see table S2 for a full description of variables). Specifically, we related year-to-year change in log collated index of abundance, *R*_*t*_, to climate variables using a generalized least squares model. We took into account temporal autocorrelation using a first-order autoregressive covariance structure. For example, a model with three climate variables

$$R_{t}=N_{t}-N_{t-1}=b_{0}+b_{1}W_{t}+b_{2}W_{t}+b_{3}W_{t}+e$$ (1)

where *N*_*t*_ and *N*_*t−*1_ represent the log collated index in the current and previous year, respectively, and *b*_1_ represents the coefficient of the climate variable (*W*) at time *t*. We allowed for lagged year effects in the models to account for direct and indirect impacts of climate on, for example, the larval and egg stages of our study species (*16*) or as a result of altered interspecific interactions or delayed density dependence (*37*). The number of possible explanatory variables used in these analyses was 24, representing the mean temperature and rainfall from the summer of the current year, backward in time to account for the previous 12 seasons, that is, up to and including autumn 2 years’ previously. Climate data for autumn of the current year were not included because UKBMS data were not collected beyond September. However, we limited the number of possible explanatory variables in each model to a maximum of three to avoid overparameterization and prevent overfitting, and tested every possible combination of variables; each species’ best model was chosen as the one with the lowest corrected Akaike information criterion (AICc).

**Quantifying species’ sensitivity and exposure to climate.** We quantified the sensitivity of each of our study species according to the amount of variation in year-to-year abundance changes that could be explained by climate. To do this, we calculated fitted *R*^2^ values from each species’ best climate model (Eq. 1), which represents the proportion of variation in the year-to-year change in species’ population index explained by climate variables (for example, see Fig. 5, E and F). Fitted *R*^2^ values were strongly correlated with *R*^2^ values obtained from an independent test of model performance (fig. S3).

Exposure encompasses both an individual species’ biological characteristics (the components of climate to which it is sensitive) and the changes in its physical environment (the amount and direction of change in those components of climate that it is responsive to). We measured exposure using each species’ best climate model (Eq. 1), which describes the components of climate the species is most responsive to. For each species, this climate model was used to model year-to-year changes in species’ abundance from 1970 to 2010, on the basis of the variation in climate over that period (which matches the time period of distribution data). Exposure was calculated as the mean predicted annual change in index, averaged over the whole time period (1970–2010; Fig. 5).

**Quantifying species’ responses to climate change.** *Changes in abundance*: Count data for each species were used to calculate annual collated indices of abundance from 1976 to 2012 (butterflies) and from 1968 to 2012 (moths). For each species, a log-linear generalized linear mixed-effects model with a fixed categorical year effect and a random site effect was applied to the annual count data; we used a random effect for site to control for variation in species’ abundances among sites. Indices were standardized before analysis (so that the mean trend per species was the same) so that they represented relative change in abundance rather than absolute change (Fig. 2). Long-term change in abundance over time was calculated as the slope of a linear model relating (log) collated index to year.

*Changes in distribution size and northern range margin*: Changes in distribution size and northern range margin were calculated for all study species between two discrete time periods (1970–1985 and 1995–2010). Time periods, rather than individual years, were analyzed to reduce the effects of interannual variability in recording effort (*38*). Unlike abundance data, recorder effort for distribution data varies considerably over time, and so we only considered locations with good recording effort in both time periods (separately for butterflies and moths), following three steps. First, for each hectad within the study area, the nearest 100 hectads with at least one record in both time periods were identified—hereinafter termed “neighborhoods” (fig. S4). Second, the total number of unique species recorded within each neighborhood was calculated. Third, each focal hectad was classed as “well-recorded” if at least 10% of the species in the neighborhood of each focal square were observed within it (fig. S2). This assessment of a good recording effort established an equivalent threshold of effort across GB (given that species richness is greater in the south). Our results remained similar if we analyzed more comprehensive (but less consistent) distributional data from less well recorded locations (fig. S2); estimated changes in absolute range size and northern range margin were strongly correlated between the “recorded” and “well-recorded” data sets (Spearman’s *r* for range size: moths, 0.84, *P* < 0.001; butterflies, 0.99, *P* < 0.001; Spearman’s *r* for northern range margin: moths, 0.78, *P* < 0.001; butterflies, 1.00, *P* < 0.001; fig. S5). All results in the paper (other than fig. S5) pertain to the well-recorded hectads.

For each species, two metrics of distribution change between the two time periods were calculated: change in distribution size (change in the number of occupied hectads per decade) and change in the location of the northern range margin, calculated as the difference between the mean latitude of the 10 most northerly hectads, in kilometers per decade (for example, see Fig. 5, A and B). The species-specific values of changes in distribution size and northern range margin were standardized before analysis to remove the influence of outlying data points and because we were interested in relative changes, rather than absolute changes, among species.

**Relating changes in species’ distributions and abundances to their sensitivity and exposure to climate.** Generalized linear mixed-effects models were used to assess distributional (standardized change in range size and northern range margin) and abundance changes in relation to species’ sensitivity and exposure to climate, allowing for an interaction between these two predictor variables. The gamlss package in *R* (*39*) was used to fit models because this package allowed for skewed error distributions. For each model, the most parsimonious error distribution was identified using the “fitDist” command—models were refitted with the next-best error distribution if they did not converge. In all but one case, models fitted using this approach were better (that is, had lower AICc’s) than equivalent models, using Gaussian error distributions (tables S3 and S4). Candidate models were identified as those within 2 AICc units of the AICc best model. Moth and butterfly analyses were kept separate because of different recording methodologies and error structures in the data sets, and preliminary analysis suggested that the relationships between species’ responses, sensitivity, and exposure for each taxonomic group were different. Although abundance trends were extracted from the same count data used to derive species’ climate models, there is not necessarily any expectation for a relationship between changes in species’ exposure and observed abundance: climate models were intraspecific and each model was independently detrended (analyzing *N*_*t*_ − *N*_*t*−1_). Furthermore, exposure and sensitivity were not significantly correlated (Fig. 3C). Thus, the detrended climate models would be unlikely to predict long-term (1970–2010) abundance trends if they were driven by changes in the environment not associated with climate. Moreover, analyses of distribution change were derived from independent data sets, yet produced similar conclusions about the role of exposure, further supporting the robustness of our findings.

There was a significant positive correlation between the prevalence (number of sites each species was recorded during the UKBMS or RIS surveys) and the sensitivity of moths (*r* = 0.19, *t*_129_ = 2.23, *P* = 0.03) and butterflies (*r* = 0.40, *t*_22_ = 2.04, *P* = 0.05), which most likely reflects improved explanatory power for species with the most robust observation data. However, when accounting for species’ prevalence in models relating changes in species distributions and abundances to their sensitivity and exposure to climate, coefficients were of similar magnitude and in the same direction as models not accounting for species’ prevalence (table S5). Moreover, the proportion of variation explained by these models differed by only a few percent from those described in Table 1, with the exception of the model explaining changes in butterfly distribution sizes; the addition of species’ prevalence in this model increased the proportion of variation explained from 0.53 to 0.78 (table S5). We have taken a cautious approach in presenting the models with lower explanatory power in the main text.

## SUPPLEMENTARY MATERIALS

Supplementary material for this article is available at http://advances.sciencemag.org/cgi/content/full/1/9/e1400220/DC1 Fig. S1. Variation in the strength and direction of climate coefficients in moth (*n* = 131; A) and butterfly (*n* = 24; B) species’ best climate models. Fig. S2. Maps showing the spatial variation in recorder effort across GB, for butterfly (A) and moth (B) recording schemes. Fig. S3. Significant, positive correlation between independent and fitted *R*^2^ from each species’ climate model relating annual change in abundance trends to climate variables (Pearson’s *r* = 0.86, *t*_153_ = 21.11, *P* < 0.0001). Fig. S4. Map showing the spatial arrangement of neighborhoods around two example focal hectads (black stars). Fig. S5. Correlations between distribution changes calculated using two different levels of recorder effort. Correlations between normalized (A) range size change (Spearman’s correlation: *r* = 0.87, *P* < 0.001) and (B) distribution margin change (*r* = 0.81, *P* < 0.001) for 155 species (moths, *n* = 131; butterflies, *n* = 24) using recorded and well-recorded hectads. Table S1. Moths and butterflies (“But.”) included in the analyses. Table S2. Pearson’s correlations between climate variables. Table S3. Shapiro tests for normality of residuals and error distributions of candidate models in Table 1. Table S4. Candidate models (within 2 AIC units of the best model) for multivariate regressions relating response variables to the sensitivity (“Sens”) and exposure (“Exp”) of moths (*n* = 131) and butterflies (*n* = 24) to climate. Table S5. Candidate models (within 2 AIC units of the best model) for multivariate regressions relating response variables to the sensitivity (“Sens”) and exposure (“Exp”) of moths (*n* = 131) and butterflies (*n* = 24) to climate, including species’ prevalence as an additional predictor.
